# Persistent Homology-Based Topological Analysis on the Gestalt Patterns during Human Brain Cognition Process

**DOI:** 10.1155/2021/2334332

**Published:** 2021-11-01

**Authors:** Zaisheng Liu, Fei Ni, Rongpeng Li, Honggang Zhang, Chang Liu, Jiefang Zhang, Songyun Xie

**Affiliations:** ^1^College of Information Science and Electronic Engineering, Zhejiang University, Zheda Road 38, Hangzhou 310027, China; ^2^Communication University of Zhejiang, Hangzhou 310018, China; ^3^Northwestern Polytechnical University, Xi'an 710129, China

## Abstract

The neuropsychological characteristics inside the brain are still not sufficiently understood in previous Gestalt psychological analyses. In particular, the extraction and analysis of human brain consciousness information itself have not received enough attention for the time being. In this paper, we aim to investigate the features of EEG signals from different conscious thoughts. Specifically, we try to extract the physiologically meaningful features of the brain responding to different contours and shapes in images in Gestalt cognitive tests by combining persistent homology analysis with electroencephalogram (EEG). The experimental results show that more brain regions in the frontal lobe are involved when the subject perceives the random and disordered combination of images compared to the ordered Gestalt images. Meanwhile, the persistence entropy of EEG data evoked by random sequence diagram (RSD) is significantly different from that evoked by the ordered Gestalt (GST) images in several frequency bands, which indicate that the human cognition of the shape and contour of images can be separated to some extent through topological analysis. This implies the feasibility to digitize the neural signals while preserving the whole and local features of the original signals, which are further verified by our extensive experiments. In general, this paper evaluates and quantifies cognitively related neural correlates by persistent homology features of EEG signals, which provides an approach to realizing the digitization of neural signals. Preliminary verification of the analyzability of human consciousness signals provides reliable research ideas and directions for the realization of feature extraction and analysis of human brain consciousness cognition.

## 1. Introduction

In recent years, with the development of neural networks, researchers are committed to explaining the intrinsic nature of human consciousness generation and artificial intelligence (AI). One of the research directions is to explore the laws of human brain cognition and consciousness generation process to promote the development of machine learning technology. In communication technology, the realization of brain-to-brain communication (B2BC) under the support of future 6G technology also urgently needs a method to realize the digitization of human brain nerve signals to support the development of its research. The most typical analysis method of electroencephalogram (EEG) signals is based on the brain signals' characteristics by filtering, artifacts removing, event-related potentials (ERP) analysis, and brain domain heat map with respect to the original time-domain signals. The complex and dynamic multichannel time-domain signal is not an ideal carrier for information transmission. Currently, various digital analysis methods based on the EEG signals are constantly being proposed and improved [1–4], such as single-trial analysis and other diverse methods, which take into account the significant differences in EEG signals between different subjects. Furthermore, [3] attempts to extract the digital features that may be more relevant and simpler regarding the signal, which coincides with the first step of B2BC: the digitization process of neural signals. Combining the relevance enlightenment of B2BC and AI, the analysis of the human brain's cognitive process is of forward-looking value.

Gestalt psychology theory is the pioneering foundation of modern cognitive learning theory, which was established in the early twentieth century by psychologists Westheimer W. Kohler and K. Koffka based on similitude study [5]. They believe that thinking is a holistic and meaningful perception rather than a simple collection of connected representations and argue that learning lies in forming a gestalt, which aims to change one gestalt into another. This cognition process is fundamentally different from the current image recognition model of deep learning empowered by artificial neural networks (ANNs).

At present, with the rapid development of deep learning, newer and stronger algorithm models emerge endlessly, and their computing power and learning ability for specified tasks become increasingly powerful. On top of this basis, some researchers initiate ambitious new goals and turn to focus on making AI more “intelligent,” that is, achieving brain-like intelligence. They expect machine learning to achieve what the human brain can do and solve problems or recognize things like the human brain. It is well known that conventional neural networks are designed by the inspiration of the fundamental principle of signal transmission in a single nerve cell. Therefore, the linkage nature of the whole biological neural network is the direction we need to explore as the next frontier. It can inspire us to build brain-like intelligence and transfer from the traditional machine learning process to a more advanced consciousness level. By exploring the act of brain cognition, it is potentially possible to probe into the generation of consciousness [6], not limited to what kind of consciousness the brain produces.

Researchers have made attempts to explore neural networks and the human brain's biological patterns [7–15]. To gain insight into the brain's response to external stimuli, scientists have developed functional network analysis methodology because they assert that brain functionality is determined by the internal interaction between different neurons as well as different brain regions [11]. They set out to analyze the neural signals displayed by the brain as a whole. The spatial and connective relationship of neurons within the brain structure is a complex connection model, which has been used to analyze the human brain's activity with topological tools for a long time. The initial focus of this kind of research is on the somatosensory sensations (e g., hot and cold sensations and pain sensations) that are easy to recognize in brain signals [12]. Afterward, abnormal EEG responses (epilepsy seizures) [13], steady-state visually evoked potential (SSVEP), movement intention detection [14], and emotion classification [15] were analyzed. We compared the results obtained by various EEG analysis methods in various fields. Among them, the detection accuracy of schizophrenia reached a balanced accuracy of 89.59%; the detection of moving images reached a recognition rate of 64.9%–79.5%; and the classification of emotional EEG signals based on gender reached 90.4% (SVM) and 92% (KNN) [16].

In particular, inspired by the recent research on Gestalt recognition for which Baker et al. [17] and Been Kim et al. [18] provided totally conflicting conclusions, the discussion on the differences between artificial neural networks and the human brain cognition process has motivated us to follow research on the cognitive process at the level of consciousness. Nevertheless, it is well realized that the human brain's cognition on the overall outline of geometric patterns faces local and global problems in the previous Gestalt experiments.

The mathematic tools of algebraic topology are uniquely equipped to provide quantitative information about both the local and global properties of an arbitrary graph [8]. Accordingly, topological data analysis (TDA) is capable of providing a series of new topological and geometric methods to analyze the brain's neural networks covering EEG signals, among which persistent homology is one of the key approaches. [19–24]. Persistent homology analysis provides efficient algorithms for calculating the Betti number of each complex graph in the network families under consideration and encodes the evolution of the nested complex homology groups at different networking scales. Consequently, it helps understand the EEG data better and keeps analytical stability concerning perturbations or noise in the EEG signals.

In our study, 20 participants were considered in traditional visual stimulation experimental methods and collecting EEG signals at the same time. The neurophysiological evaluation of the contour in the Gestalt experiment was investigated by exploiting Euler characteristics and persistent homology features of the EEG signal. On that basis, how the regions of the brain are involved in contour recognition was interpreted by selecting Vietoris–Rips filtration.

The main contributions of this work are as follows:

1. The topology calculation method adopted in this experiment provides effective separability of the EEG signals of contour cognitive behavior and realizes the digital feature extraction of EEG signals
2. We provide reference significance and a reference method for B2BC and other work that needs to realize the digital feature extraction of EEG signals
3. We demonstrated the feasibility of using persistent homology modeling to analyze EEG signals

## 2. Experiments and Methods for Assessing Brain Cognition's Gestalt Patterns

The general framework for the neurophysiological assessment process and method of Gestalt contour cognition is illustrated in Figure 1, which is based on topological data analysis enabled by persistent homology. During the brain cognition process, subjects first watch random sequence diagram (RSD) pictures repeatedly at fixed intervals and then watch Gestalt (GST) images in the same manner. Meanwhile, the EEG data are collected by a special cap with sensing electrodes synchronously (Step I). Then two methods are used for calculating the correlation coefficient: one is to calculate the phase correlation coefficient (0–1) of the EEG signals between the sensors through the algorithm based on Hilbert transform to construct the correlation matrix and the other is to calculate the standardized Euclidean distance between the sensors to construct a distance matrix (Step II) [13] for obtaining the topological Vietoris–Rips simplex (Step III). Finally, persistent homology methodology is applied to analyze the brain's neurophysiological features stimulated by various pictures across different qualities (Steps IV and V).

### 2.1. Stimuli

As shown in Figure 2, we have selected two representative types of Gestalt pictures with the existence and nonexistence of a specific outline of a standard triangle. One is the picture of GST that people can easily recognize the outline of the triangle, and the others are the pictures of RSD. The size and quality of the two types of pictures are the same, and both are 1,440 × 1,080 resolution. To explore the characteristics of changing consciousness in a subject's cognition process, we repeat the RSD 30 times and then repeated the GST 10 times to increase the samples' amount and eliminate potential experimental errors.

### 2.2. Procedure

After a general introduction to the experiment and the EEG cap preparation, the subjects start the test with EEG recording, which is described in Figure 3. The EEG recordings of two cognition periods correspond to two continuous stages in the whole process. The first stage is to collect the EEG signals when the subject does not have a clear cognition of RSD, and the second stage is to collect the signals when the subject recognizes the outline of the triangle from the GST. When the subjects start to identify the triangle's intrinsic outline from the GST, each trial began with a fixed time slot that lasts 1 second, and then the RSD or GST image appear for 10 seconds. After that, a rest time slot appears to remind the subjects that they could take a break for 1 second. One by one, the subsequent trials start to run.

### 2.3. Subjects and Equipment

The EEG data are measured from 20 healthy volunteers (9 males and 11 females, in the age group 19–27) with normal (or corrected to normal) vision. Volunteers are mainly sophomores and juniors. The main age group is 22 years old, with an average age of 22.4 and a standard deviation of 1.71. The experiment equipment is a standard Neuracle 64 System, which includes a 64-channel adult-sized head cap with the sensor array, EEG recorder with EEG acquisition software, and amplifier (NSW364). The sampling rate is 1,000 Hz for the EEG signals, and the filtering window is changed with frequency from 0.3 to 100 Hz.

### 2.4. Topological Data Analysis for EEG Data

Topological data analysis for the EEG data has been summarized in Figure 1, and the following provides the corresponding details.

#### 2.4.1. EEG Signals Acquisition and Preprocessing

The EEG data are collected by the EEG cap and downsampled to 250 Hz. Filtered EEG signals of different wavebands are obtained by a set of filters, including *δ* band (1–3 Hz), *θ* band (4–7 Hz), *α* band (8–13 Hz), *β* band (14–30 Hz), and the whole band (1–45 Hz).

The specific operations are as follows: during the entire acquisition process, we mark the EEG signals corresponding to different events to facilitate subsequent trial segmentation. Since the entire acquisition process is continuous, considering the activity frequency of the human brain under normal conditions, we first perform (1–45 Hz) filtering on the entire time-domain signal and then try segment to extract the target data we need, based on this perform subsequent data adjustments such as baseline calibration and downsampling.

The filtered signals from each electrode of the EEG cap correspond to a set of measuring points G. As explained before, two data analysis methods are used for characterizing the brain cognition process: one is to calculate the correlation matrix through the real-time phase relationship and the other is to define the distance matrix for each point through the signal-level correlation.

#### 2.4.2. Correlation Matrix Computing

The calculation steps are as follows:

(1) After the key feature extraction and preprocessing of the EEG signals, we get the signal of each trial period as follows:
  (1) $$\begin{array}{c} F_{\text{EEG}}=\;\left[\begin{array}{ccc} f_{11} & \cdots & f_{1N}\\ \vdots & \ddots & \vdots \\ f_{M1} & \cdots & f_{MN} \end{array}\right], \end{array}$$
where *N* is the total data length, which is equal to the sampling rate multiplied by the measurement time, and *M* is the total number of electrodes that collect the EEG signals. Each row in the matrix *F*_EEG_ represents the signals collected by one electrode.
(2) Hilbert transform [25] is performed on each signal in *F*_EEG_, that is, each row, to obtain a new matrix *H* (*F*_EEG_).
(3) *H* (*F*_EEG_) obtained by step 2 is used to calculate the instantaneous phase of each electrode:
  (2) $$\begin{array}{c} \phi =\arctan\left(\frac{\text{H}\left(F_{\text{EEG}}\right)}{F_{\text{EEG}}}\right). \end{array}$$
(4) The value of the corresponding element of the incidence matrix is calculated by equation (3). The absolute value is taken and then combined to obtain the incidence matrix equation (4):
  (3) $$\begin{array}{c} C_{pq}=\left\{\begin{array}{cc} \frac{1}{N}\left|\overset{N}{\underset{n=1}{\sum }}\exp\left(j\left\{\phi^{p}\left(n\right)-\phi^{q}\left(n\right)\right\}\right)\;\right|, & p\neq q,\\ 0, & p=q, \end{array}\right) \end{array}$$
  (4) $$\begin{array}{c} C_{M\times M}=\left[\begin{array}{ccc} C_{11} & \cdots & C_{1M}\\ \vdots & \ddots & \vdots \\ C_{M1} & \cdots & C_{MM} \end{array}\right], \end{array}$$
where *j* is an imaginary unit and *ϕ*^*p*^(*n*) and *ϕ*^*q*^(*n*) represent the *n*-th instantaneous phase in the electrode *p* and *q*, respectively.

#### 2.4.3. Distance Matrix Computing

The filtered signal from each electrode in the EEG cap constitutes a set of sampling points *G*, and the distance between electrodes with different channels is calculated by [13]

(5) $$\begin{array}{c} d\left(r,t\right)=\sqrt{\overset{N}{\underset{k=1}{\sum }}{\left(\frac{{r|}_{k}}{s_{k}}-\frac{{t|}_{k}}{s_{k}}\right)}^{2}}, \end{array}$$

where *r|*_*k*_ and *t|*_*k*_ stand for the *y*-component of different electrodes in (*x*_*k*_, *y*_*k*_) and *s*_*k*_ is the sample standard deviation calculated from all *y*-components at position *k* in channel *r*.

#### 2.4.4. Simplicial Complexes Construction

Simplicial complexes are constructed by Vietoris–Rips filtration according to either the correlation matrix or the distance matrix obtained in Step II, which is illustrated in Figure 4.

#### 2.4.5. Euler Characteristics

Before calculating the persistent entropy, we supplement Euler entropy to do a preliminary analysis of the separability of the topological properties of the data, which also provides a basis for the persistent homology separability. The topological structures of original EEG signals are constructed by Vietoris–Rips filtration: one uses the phase-locked value (PLV) of the EEG signals data as the normalized correlation coefficient (*C*-matrix) between electrodes and the other uses the level correlation distance as the normalized correlation coefficient (*D*-matrix). Euler entropy can be calculated according to the Betti numbers. In the process of Vietoris–Rips filtration, the Betti numbers change all the time, so we can restore an Euler entropy curve. The Euler entropies of brain networks for different values of *e* are calculated, and it is a remarkable fact that Euler entropy has a negative peak with the change of *ε*. Since the *ε* value corresponding to the negative peak of Euler entropy is different between the clear and unclear situation, we further calculate the *ε* value when the negative peak of Euler entropy appears, which is taken as a phase transition point in this work. In the topological modeling of human brain structure, the phase transition point is shown by Euler entropy often represents a critical point change in brain activity [8].

#### 2.4.6. Persistent Homology Analysis

Persistent homology is an algebraic topology methodology that counts the number of *n*-dimensional holes in a topological space, that is, Betti number. The Betti number of a generic topological space *S* is composed of *β*_0_, *β*_1_, and *β*_2_ in this paper. *β*_0_ is the number of connected components in *S*; *β*_1_ is the number of holes in *S*; and *β*_2_ is the number of voids in *S*. During the filtration, the time when a *k*-dimensional hole appears in the simplicial complex is recorded as *T*_start_, while *T*_end_ is the time when the *k*-dimensional hole disappears. Accordingly, the *k*-dimensional Betti interval is defined by [*T*_start_,  *T*_end_], and the corresponding persistence barcode is its graphical representation of it [8, 26, 27]. On the other hand, persistent entropy (PE) provides a new entropy measure to extract the feature of topological space by persistence barcode. In this paper, *B*={(*x*_*i*_, *y*_*i*_)*|iεI*} is set to the persistent barcode group associated with the filtration of topological space *S*, where *i* is a set of indexes (Figure 5). Accordingly, the persistent entropy H of the simplicial complex filtration is calculated by the following equation:

(6) $$\begin{array}{c} H=-\sum_{i\varepsilon I}p_{i}\log\left(p_{i}\right), \end{array}$$

where *p*_*i*_=*y*_*i*_ − *x*_*i*_/*L* and *L*=∑_*iεI*_(*y*_*i*_ − *x*_*i*_). Moreover, *H* can be rescaled, and $\hat{H}$ is treated as the persistent homology feature of the EEG data in this paper and expressed as follows:

(7) $$\begin{array}{c} \hat{H}=\frac{H}{\log\;\ell_{\max}\;}, \end{array}$$

where *ℓ*_max_ is the maximum interval in the considered persistent barcode group.

Topological patterns of the EEG data evoked by the RSD/GST pictures are constructed by Vietoris–Rips filtration, as shown in Figure 6. To examine the relationship between different brain regions and the perception of image shape and contour, the EEG mapping results are supplemented and drawn in Figure 6. When the subjects perceive irregularly distributed images, more brain regions are involved, with nonprominent features, but when they perceive ordered images, there will be clear reaction areas with more prominent features. Therefore, we hypothesize that vague cognitive goals make the task more difficult and lead to more mental activities. In addition, due to the intense brain activity observed in the frontal lobe, the frontal lobe's function needs further investigation. The frontal lobe is the physiological basis of the most complex mental activities. It is responsible for planning, regulating, and controlling human mental activities, which plays a vital role in human's advanced and purposeful behaviors. Figure 6 indicates the correlation between human perception of shapes and higher-level cognitive processes covering Gestalt patterns. These results verify our method's effectiveness in describing the intrinsic correlation between the EEG signals and shape cognition, and our method is closer to the actual biological response process.

In this regard, our preliminary Euler entropy analysis diagram is shown in Figure 7. The two types of calculated Euler entropy show the difference in their phase transition points. The red line represents the RSD in the state of unclear recognition, and the blue line represents GST that can recognize the outline of a triangle. It can be seen that the phase transition point of the GST sample will appear earlier than the RSD. The data result of the overall sample is shown in Figure 8.

## 3. Result and Discussions

It can be observed from Figure 8 that the phase transition point of GST trials of most samples is before the RSD, which intuitively shows the separability of the overall topological characteristics of the whole brain signal, so further continuous coherence analysis can be carried out on this basis.

To reduce the computation time of analyzing topological features, the change of persistent entropy of the subjects at different time latencies after the picture appearance is investigated first. There is a difference between the RSD and GST trials. Without being informed of the experiment's purpose, the subjects observed the RSD pictures first, which are disorderly and random. Accordingly, the overall EEG levels are shown in each trial. They were all at a certain level in a relatively balanced manner, while regarding the GST pictures, it was intuitively reflected within 2 s, and the EEG level was stable afterward. Therefore, the EEG signals of two seconds after displaying the image are selected for the persistent homology analysis in this paper.

Table 1 shows the range, mean value, and maximum value of the distinguishing degree of the two types of cognitive behaviors investigated by adopting persistent entropy as the overall experiment's discrimination standard. The average distinguishing rates of each frequency band classified by *C*- and *D*-matrix were all greater than 70%, and the optimal distinguishing rates reached 90% and 85% for *C*- and *D*-matrix, respectively.

Figure 9 shows the respective performance and comparison of the persistent entropy obtained by the two different matrix calculation methods. The blue line represents the participants' response to GST, and the red line represents their response to RSD. Based on the statistical classification of the 20 subjects and the frequency comparison, it is clear that both methods clearly describe the separation feature in terms of persistent entropy between the two topological patterns in the two types of brain cognition situations. We further draw a comparison chart of the GST and RSD values calculated by the correlation matrix as shown in Figure 10. According to Figures 9 and 10, almost all the persistent entropy values for the topological structure of the EEG signals induced by GST (blue) are higher than that induced by RSD (red); the opposite is the case when the persistent entropy is calculated by the distance matrix. From the measurement and analysis results, it is evident that the bands with significant differences are the *α* and *θ* bands, which are in line with the corresponding trend of the overall original signal. However, in the *β* band, the properties of the two types of methods are similar, and the results of the comparison of RSD and GST are similar as depicted in Figure 11.

As a summary, we have proposed a neurophysiological approach for cognitive assessment of the shape and contour of the Gestalt images via EEG. When the subjects perceive RSD images, compared with the GST image, more brain regions are involved in the cognition process. It can be understood that the human brain is in a state of randomness in this case. TDA is used to extract the physiological features of EEG signals induced by the shape contours. The results verify that the EEG data induced by the GST image are in the beta band, and the persistent entropy values obtained by the two calculation methods are lower than that of the RSD image. The persistent entropy values in the *α* and *θ* bands and the overall 1–45 Hz band consistently show that *PE*_GST_ > *PE*_RSD_ with the correlation matrix calculation method and *PE*_GST_ < *PE*_RSD_ with the distance matrix calculation method.

Compared with the conventional neurophysiological methods based on evoked potentials (requiring a specific experimental paradigm), our approach provides a generalizable method that can extract the overall information from the whole brain signal, not just the characteristic performance. Our approach focuses not only on the brain response to external stimuli but also on the algorithms designed to normalize and extract numeric features that can be reliably classified and represent different cognitive perceptions. The algebraic topology is used to explain the coordination relationship between various neural regions in the human brain. This work can serve as an inspiration for the analytical approach to the collaborative work of complex neural networks. The dimensionality of the complex neural network model is reduced to one-dimensional persistent entropy to measure its characteristics.

Since this paper focuses on a specific case of Gestalt contour cognition, future research may extend to more analysis of different Gestalt contour cognitions and even color or content cognition and progressively try to leverage TDA to explain the cognitive process. Unlike the previous EEG signal analysis experiments, this work implies the feasibility to interpret the human brain consciousness patterns in a divisible manner, and it is a preliminary exploration from feeling to consciousness. Furthermore, the deepening grasp of the brain neural network's linkage behavior in the brain response process from external stimuli to digital features may inspire us to build a new artificial neural network structure, which requires further research and experimentation.

## 4. Conclusions and Future Work

In this paper, we have proposed an approach physiological evaluation of contour cognition from EEG by using persistent homology of brain network and extracted its separable digital feature, persistent entropy (PE). Our approach has acquired cognitively related neural information via integrating the EEG collection with the traditional Gestalt psychology test procedure and obtained physiologically meaningful features of brain responses to different shape outlines by topological data analysis (TDA). The validation experiment results show that when subjects perceive chaotically distributed images, more brain regions are involved, but the level values are more average, and when they perceive ordered images, there will be clear reaction areas with more prominent features. The PE calculated by using two different EEG correlation feature extraction matrices is all separable. In the *α*, *θ*, and (1–45 Hz) bands, the overall performance is consistent, and the two types of calculations in the *β* band have reached a unified result of the calculated value and the classification situation. The above results can intuitively show that in some specific B2BC interaction scenarios, the transmission of a specific human brain nerve signal into a characteristic signal (PE) can be achieved.

The neurophysiological assessment process of Gestalt contour cognition is a preliminary study to explore human consciousness formation. The experimental results show that the conventional EEG signal can be digitized and converted into the matrix relationship between the electrode points, and then the Vietoris–Rips complex is constructed to use the topological calculation to express the characteristics. It encouragingly shows good separation, which provides a possibility for the development of B2BC.

At present, there still exist some limitations to be addressed, specifically in the following two aspects:

1. One is that noninvasive EEG acquisition equipment cannot completely restore the spatial location generated by electrical signals, which means that the accuracy of our topological reconstruction construction cannot restore the original signals generated by consciousness
2. Second, the use of algebraic topology is still in the preliminary stage, and more experiments are required to verify the robustness of the method.

The outlook for future work can be expanded from two dimensions of breadth and depth. The breadth is that there are many forms of conscious thinking because the project is an exploratory experiment, and we use contour recognition as the starting point. Subsequent work can be developed to the consciousness analysis of more advanced cognitive behaviors, such as the calculation of simple mathematical problems, the judgment of the right and wrong of simple logic, and so on. The depth requires us to further enhance and strengthen this method on the basis of existing research. We can try to refine the research based on gender differences, brain region selection, more detailed trial segmentation, and frequency band selection to verify the robustness and reliability of the method proposed in this paper. The realization and gradual advancement of these tasks will lay a solid foundation for our future realization of brain-computer interconnection and brain-to-brain interconnection technology, and this is also an effective means to simulate and realize human intelligence. The analysis of human consciousness and thinking activities in this work also expands the breadth and depth of EEG analysis. The research in this area is still in the preliminary stage for the time being, and we provide enlightening significance for reference.

## Figures and Tables

**Figure 1:** The neurophysiological process and method of Gestalt contour cognition with topological data analysis.

**Figure 2:** Two types of Gestalt pictures used for the brain cognition experiments: GST and RSD.

**Figure 3:** The procedure of Gestalt pattern cognition.

**Figure 4:** Vietoris–Rips filtration in persistent homology-based topological data analysis.

**Figure 5:** Persistent barcode group.

**Figure 6:** EEG mapping and the corresponding Vietoris–Rips simplex. Red indicates high levels of neuronal activation in EEG mapping.

**Figure 7:** Phase transition points in Euler entropy curve.

**Figure 8:** Comparison of phase transition points by C- and D-matrix.

**Figure 9:** Comparison of persistent entropy calculated by C- and D-matrix (1).

**Figure 10:** Comparison of persistent entropy calculated by C- and D-matrix (2).

**Figure 11:** Beta bands.

**Table 1:** The table of distinguishing accuracy.

	Distinguishing rate range (%)	Average (%)	Max (%)
*C*-matrix	65–90	73.33	90
*D*-matrix	55–85	71.67	85

## Data Availability

The data in this study are collected by our own experiment and are available from the first author (liuzs@zju.edu.cn) upon request.
